RETRACTED

# Recognition of Key Genes in Human Anaplastic Thyroid Cancer via the Weighing Gene Coexpression Network

**DOI:** 10.1155/2022/2244228

**Published:** 2022-06-23

**Authors:** Yun Gong, Fanghua Xu, Lifei Deng, Lifen Peng

**Affiliations:** ^1^Health Management Center, Jiangxi Provincial People's Hospital (the First Affiliated Hospital of Nanchang Medical College), Nanchang, Jiangxi 330006, China; ^2^Department of Pathology, Pingxiang Hospital Affiliated to Southern Medical University, Pingxiang, Jiangxi 337000, China; ^3^Department of Head and Neck Oncology, Jiangxi Cancer Hospital, Nanchang, Jiangxi 330029, China; ^4^Department of Otolaryngology Head and Neck Surgery, Jiangxi Provincial People's Hospital (the First Affiliated Hospital of Nanchang Medical College), Nanchang, Jiangxi 330006, China

## Abstract

**Methods:**

For determining pathways and key genes that have relation with development of ATC, differentially expressed genes (DEGs) from GSE33630 as well as GSE65144 expression microarray were screened. Furthermore, we also worked on carrying out the task of constructing a protein-protein interaction (PPI) network and the work of weighing gene coexpression network (WGCNA). DAVID was utilized for the performance of the Gene Ontology (GO) as well as KEGG pathway enrichment analyses for DEGs. We used TCGA THCA data and GSE53072 to further verify the hub gene and hub pathway.

**Results:**

We came to the conclusion of the recognition of a total of 1063 genes as DEGs. Analysis regarding functional and pathway enrichment showed that there existed a notable enrichment of upregulated DEGs in the organization of extracellular structure and matrix organization, as well as in organelle fission and nuclear division. The downregulated DEG was markedly gathered in the thyroid hormone metabolic process and generation, as well as in the metabolic process of cellular modified amino acid. We identified 10 hub genes (CXCL8, CDH1, AURKA, CCNA2, FN1, CDK1, ITGAM, CDC20, MMP9, and KIF11) through the PPI network, which might be strongly linked to the carcinogenesis and the development of ATC. In the coexpression network, 6 modules that were relevant to ATC were recognized. The modules were related to the interaction of signaling pathway of p53, Hippo, PI3K/Akt, and ECM-receptor. This hub genes and hub pathway were further successfully validated as a potential biomarker for carcinogenesis and prediction in another database GSE53072.

**Conclusion:**

To summarize, this research displayed an illustration of hub genes and pathways that had relation with ATC development, which suggested that DEGs and hub genes, recognized on the basis of bioinformatics analyses, were valuable in the diagnosis for patients with ATC.

RETRACTED

## 1. Introduction

Thyroid cancer, the commonest malignancy that is related to endocrine, occupies a proportion above 90% of endocrine cancers [1]. Thyroid tumors are mostly cancers that are differentiated in terms of pathology and display good prognosis with a survival rate in the amount of time of five years higher than 98% [2]. Of these kinds of differentiated thyroid cancers (DTC), the commonest kind belongs to papillary thyroid cancer (PTC), which occupies a percentage of around eighty in all of the thyroid cancers. Among the entire thyroid malignancies, carcinoma of follicular thyroid and papillary thyroid occupies around a percentage of ninety [3]. Nonetheless, the most fatal histotype belongs to anaplastic thyroid cancer (ATC), with a five-year survival rate being merely around 8%. This type of cancer is undifferentiated and almost incurable with an approximate six-month median survival rate, which accounts for an essential proportion of deaths that are relevant to thyroid cancer [4]. Due to the gloomy prognosis, it contributes to a percentage during forty to fifty in the entire amount of deaths that have relation with thyroid cancer in the country of America. Therefore, it is essential to gain a deep knowledge of ATC etiology in terms of its molecular foundation [5]. In spite of a rising number of researches revealing that genetic mutations play a role in ATC, the molecular mechanism underlying ATC progression remains unclear [6]. Nevertheless, the priority is still to identify novel therapeutic biomarkers or targets for ATC prognosis, diagnosis, or prediction.

At present, the association between genes and the progression of ATC has been identified with gene expression profiles [7]. At the same time, a number of researchers also adopted an integrated approach for the purpose of screening changes in ATC [8, 9]. Nevertheless, the majority of studies only placed emphasis on filtering differentially expressed genes. Although similarity of genes in expression patterns means that they are probable to be associative in function, the ignorance of high-degree interconnection between genes remains to be an issue. The weighted gene expression network analysis (WGCNA), which is given the definition as a method of systems biology, gives a description of genes across microarray or RNA sequence data in terms of the correlation patterns that are among the genes. Besides, this method, viewed as an algorithm, serves the purpose of not only seeking clusters (modules) of genes that are highly correlated and also for recognizing genes clusters or modules that are related to phenotype [10]. In this research, an attempt is made for the first step of filtering DEGs, construction of interaction networks of protein-protein as well as a coexpression network in terms of relationships that are between genes via the method of systems biology which is on the basis of the WGCNA. And it is also meant to assist the recognition of key genes as well as pathways that have relation with ATC's carcinogenesis.

RETRACTED

## 2. Materials and Methods

### 2.1. Data Acquisition

The original expression profile datasets that make a comparison with ATC and normal thyroids tissues in the aspect of gene expression were provided by GEO databases (http://www.ncbi.nlm.nih.gov/geo/). GSE33630's and GSE65144's microarray expression profile datasets were obtained through the GEO database. This database is known as a public functional genomics data storage that is about aspects of microarrays, chips, and high-throughput gene expression data. Microarray data of GSE33630 [11] and GSE65144 [12] depended upon the GPL570 [HG-U133_Plus_2] Affymetrix Human Genome U133 Plus 2.0 Array. The GSE33630 dataset is available with 45 normal thyroids (NC), 49 papillary thyroid carcinomas, and 11 anaplastic thyroid carcinomas. The GSE65144 dataset contains 12 anaplastic thyroid carcinomas and 13 normal thyroids samples. Based upon the annotation information that was obtained through the platform, the further step was carrying out the work of the transformance of corresponding gene symbols from probes. For validation, the work of downloading and analyzing The Cancer Genome Atlas (TCGA) [13] (https://cancergenome.nih.gov/) thyroid cancer data, and GSE53072 [14] was performed as the next step.

### 2.2. DEG Screening

First of all, the originally obtained data of expression were undergoing quartile data normalization and background correction. For the next step, through the assistance provided by robust multiarray average (RMA) in the R Affy package, the data were changed into expression measures. For the further step, the “limma” R package was performed as the assistance of recognizing differentially expressed genes (DEGs) between anaplastic thyroid carcinoma's and normal thyroid's samples [15]. |log2*FC*| ≥ 2 and *P* value < 0.01 were both regarded as being of statistical significance for the DEGs. A heat map of the sample was constructed, and the DEGs were identified utilizing the pheatmap software package of the R software functional and pathway enrichment analysis. Utilizing the edgeR package, DEG screening was carried out for TCGA data. According to the Benjamini-Hochberg (BH) procedure, the choice of *P* < 0.01 as well as absolute log2FC > 2 being the cut-off criteria was made.

### 2.3. Gene Ontology's and KEGG Pathway's Enrichment Analysis

The Database for Annotation, Visualization and Integrated Discovery (DAVID; https://david.ncifcrf.gov/) (version 6.8), given the definition of an information database in terms of biology that serves on the Internet, offers functional annotation information of genes in the form of a comprehensive set. Besides, it is also an analysis tools to researchers for obtaining the knowledge of gene biological meaning. Gene Ontology (GO) enrichment analyzes common DEGs for biological process (BP), cellular component (CC), and molecular function (MF) terms via assistance offered by utilizing DAVID [16, 17]. Kyoto Encyclopedia of Genes and Genomes (KEGG) is given the definition of an online database resource that assists in comprehending biological systems and high-level functions from massive-scale molecular datasets that can be gained from high-throughput experimental technologies. DEGs' signaling pathway analysis was carried out against the KEGG pathway database through assistance given by utilizing DAVID [18]. Merely the pathways that have more than two gene hits and *P* < 0.05 (Benjamini-Hochberg procedure) were demonstrated.

RETRACTED

### 2.4. Analysis of the Protein-Protein (PPI) Interaction Network

The Search Tool for Retrieval of Interacting Genes (STRING; https://string-db.org/cgi/input.pl) (version 10.0) database, given the definition as an online database of biology, is used for collecting comprehensive information on proteins for the purpose of evaluating the associations that are direct (physical) and indirect (functional) [19, 20]. In the current research, the STRING database was utilized to achieve the construction of the DEGs' PPI network. An interaction that had a score > 0.4 in combination was regarded as being statistically significant. Then, analysis was completed through the application of the STRING database, and the Cytoscape software was utilized for visualization. Cytoscape (version 3.6.0), known as a bioinformatics software, serves the purpose of performing computational analysis of the emerging cellular network as well as merging the experimental omics datasets [21]. Furthermore, this software also serves the purpose of constructing DEGs' PPI network. The molecular complex detection (MCODE) plug-in of Cytoscape is given the definition as an app that serves the purpose of helping to cluster a given network according to topology for discovery of regions that are densely connected and to utilize MCODE for selection of most significant hub modules of PPI networks [22]. For a subsequent step, KEGG as well as GO analyses were carried out through the assistance of utilizing DAVID for genes in this module. Meanwhile, MCODE scores > 5, node score = 0.2, *k* − core = 2, and max.depth = 100 were taken to be cut-off criteria.

RETRACTED

### 2.5. Coexpression Network Construction and Module Functional Analysis

WGCNA construction was achieved by utilizing samples and genes that were good. WGCNA network construction was fulfilled by the package “WGCNA” [9]. For the very first step, employment of the gradient method served the purpose of measuring independence as well as average connectivity degree of diverse modules whose power values were not the same. Degree of independence ≥ 0.85 was set as a threshold to consider power value as appropriate [23]. While the power value was decided, the WGCNA algorithm was used to proceed with the module construction. The smallest size of genes in every coexpressed gene module was made to be the number of one hundred. Secondly, in order to judge the quality of the sample and gene, an examination of DEGs' expression data profile was carried out. As a next step, the “WGCNA” package in R underwent being utilized for construction of a coexpression network for DEGs [24]. Firstly, calculation of Pearson's correlation matrices was carried out to serve for all of the paired genes. For the next step, the construction of a weighted adjacency matrix reached the result of fulfillment with a power function *amn* = |*cmn*|*β* (*cmn* is Pearson's correlation between genes *m* and *n*; *amn* is adjacency between genes *m* and *n*). *β*, known as a soft-thresholding parameter, was capable of putting emphasis on strong correlations that exist between genes as well as penalizing weak correlations at the same time [9]. By making use of module core genes, the performance of GO and pathway enrichment analysis was completed with a satisfactory result. Information of core genes was mapped to DAVID 6.8 (http://david-d.ncifcrf.gov/). The conclusion drawn by performing the analysis of GO and KEGG underwent transformation in txt. files as well as further visualization through the R software. *P* < 0.05 was used as a cut-off to serve the purpose of defining statistical significance.

### 2.6. Hub Genes and Pathway Validation

TCGA THCA database (based on the GEPIA database, http://gepia.cancerpku.cn/index.html) as well as the GSE53072 database served as validation for hub genes and pathway. TCGA thyroid carcinoma (THCA) data included 59 normal and 512 thyroid cancers. GSE53072 dataset contains 3 pair matched anaplastic thyroid cancer and normal thyroid samples [25]. The strategy of data mining and process of GSE53072 is the same as that used in GEO data analyzing mentioned above.

### 2.7. Statistical Analyses

Mean ± SD (standard deviation) was taken as the manifestation of data, and Student's *t*-test underwent being taken advantage of to serve for achieving the result of calculating statistical significance between the two groups. The further step was the adoption of a paired *t*-test for paired samples. The SPSS 21.0 (SPSS Inc., USA) software experienced being utilized to serve for the performance of statistical analyses. *P* < 0.05 was viewed as being of importance in terms of statistics.

RETRACTED

## 3. Results

### 3.1. Identification of DEGs in ATC Tissues

Through application of the R software's “limma” package, the analyzing work was managed for gene expression profiles of GSE33630 as well as GSE65144, including the tissues of ATC and normal thyroid with the numbers of 23 and 58, respectively. After conducting gene differential expression analysis of microarray data, 1063 genes in all were recognized as DEGs, 447 genes that were upregulated and 616 genes that were downregulated in tumor tissues (Supplementary Table S1). The construction of heat map was achieved by utilizing DEGs that ranked the top 100 according to fold change (Figure 1(a)).  Figure 1(b) manifests all DEGs' volcano plot.

### 3.2. GO Term and KEGG Pathway Enrichment Analyses of DEGs

For obtaining a greater degree of enlightenment of ATC's DEGs' function, upregulated and downregulated DEGs were transformed into DAVID. A conclusion was drawn from the GO analysis results that the upregulated genes were found noticeably gathering in organization of extracellular matrix and extracellular structure, as well as in nuclear division and organelle fission. There was a significant gathering of the downregulated DEGs in the thyroid hormone metabolic process and generation as well as in cellular modified amino acid metabolic process (Figures 2(a) and 2(b)). We could stand to benefit from these significantly enriched GO terms in terms of obtaining further knowledge of the role of DEG in the development of ATC. According to the KEGG pathway enrichment analysis that underwent being carried out for all DEGs, a conclusion drawn from the results indicated that there was a marked enrichment of the DEGs in thyroid hormone synthesis, transcriptional misregulation in cancer, signaling pathway of p53, and PI3K-Akt (Figure 3).

### 3.3. Protein-Protein Interaction (PPI) Network Construction

The PPI network of overlapping DEGs had 706 nodes and 6126 edges, including 1063 differentially expressed genes, the construction of which was fulfilled by the STRING online database (Supplementary Table S2). The outcome was transferred to the Cytoscape software for the purpose of analyzing the interactions of the candidate DEG-encoding proteins in anaplastic thyroid cancer. The cytoHubba Network Analyzer plug-in from the Cytoscape software selected the top 10 DEGs with their degree and betweenness being above fourfold of the matching median values taken as the candidate hub genes, which were identified, namely, C-X-C motif chemokine ligand 8 (CXCL8), aurora kinase A (AURKA), cadherin 1 (CDH1), cell division cycle 20 (CDC20), cyclin A2 (CCNA2), cyclin-dependent kinase 1 (CDK1), fibronectin 1 (FN1), integrin subunit alpha M (ITGAM), kinesin family member 11 (KIF11), and matrix metallopeptidase 9 (MMP9) (Supplementary Table S3). Furthermore, for the sake of detecting this PPI network's notable gathering modules, performance of module analysis reached completion. The three at top were obtained with parameters that were displayed thereinafter: degree cut − off = 5, node score cut − off = 0.2, *k* − core = 2, and max.depth = 100. Viewed from the GO enrichment analysis, module 1 could be seen as strongly linked to microtubule-based movement, mitotic cytokinesis, and positive regulation of cytokinesis; module 2 was strongly associative with inflammatory response, immune response, cell chemotaxis, cell-cell signaling, and chemokine-mediated signaling pathway; module 3 went hand in hand with collagen fibril organization, cellular response to amino acid stimulus, and blood vessel development (Figure 4 and Supplementary Table S4). Regarding the KEGG pathway enrichment analysis, the main enrichment of module 1's genes was found existing in cell cycle and p53 signaling pathway; the main participation of the genes in module 2 was in the signaling pathway of chemokine, IL-17, NF-kappa B, and TNF; module 3's genes were found primarily implicated in protein absorption and digestion, PI3K-Akt signaling pathway, and ECM-receptor interaction (Supplementary Table S5).

RETRACTED

### 3.4. Weighted Coexpression Network Construction and Analysis

As a following step of quality validation that was served for GSE33630's and GSE65144's expression data matrix, Pearson' s correlation analysis showed that no samples were outliers and all anaplastic thyroid cancer samples were identified as good samples and clustered (Figure 5(a)). Next, R's “WGCNA” package underwent being utilized, and the power of *β* = 14 (scale-free *R*^2^ = 0.85) was taken to be selection for the purpose of ensuring a scale-free network (Figures 5(b) and 5(c)). Selection of *β* = 14 served the purpose of ensuring high scale independence (~0.85) and low mean connectivity (~0.0) (Figures 2(a)–2(c)). Modules' dissimilarity was made with the number of 0.2, and 8 coexpressed gene modules in all (grey, turquoise, blue, brown, green, yellow, red, and black) were recognized with a module size cut − off ≥ 100. Except for green, yellow, red, and black modules, Gene Ontology was also carried out for the other 4 modules to serve the purpose of exploring the underlying biological process that was associative with ATC. In the turquoise module, there was an enrichment of DEGs found by the researchers in the urogenital system development, ossification, and extracellular structure organization (Figure 6(a)). In the grey module, an enrichment of DEGs was discovered in catabolic process of small molecule, organic acid, and carboxylic acid (Figure 6(b)). Blue module was found DEG gathering in organization of extracellular matrix and extracellular structure, as well as organelle fission (Figure 6(c)). In the brown module, an enrichment of DEGs was found in T cell activation as well as in lymphocyte activation's and T cell activation's regulation (Figure 6(d)).  Figure 7 demonstrates a conclusion drawn that the common pathways were associative with ATC: the signaling pathway of PI3K/AKT, p53, and Hippo signaling pathway as well as ECM-receptor interaction.

RETRACTED

### 3.5. Hub Genes and Pathway Validation

Firstly, performance of validation of hub genes was completed via utilizing TCGA ATC database (based on GEPIA database) and microarray GSE53072. The results of TCGA database showed that CXCL8, CCNA2, FN1, CDK1, ITGAM, CDC20, MMP9, and KIF11 were upregulated in tumor tissues. In the meantime, CDH1 and AURKA displayed downregulation in tumor tissues, which was a result being contrasted with thyroid tissues that were in normality (*P* < 0.05) (Figure 8). Results of GSE53072 microarray showed that there was a higher expression of CXCL8, AURKA CCNA2, FN1, CDK1, ITGAM, CDC20, MMP9, and KIF11 in ATC than normal thyroid tissues, except for the low expression of CDH1 in ATC (Figure 9).

## 4. Discussion

Anaplastic thyroid cancer (ATC), known as an unusual type divided under thyroid cancer that has a fatality rate of nearly 100%, is included in the most aggressive cancers that have ever been found in mankind. On account that ATC is uncommon, clinical experience and published case series are taken as the basis of the management of ATC patients [26]. The development of ATCs into inoperable and metastatic tumors is of frequent occurrence, and conventional treatment for ATC remains an unsuccessful method for preventing the progression of ATC [27]. In spite of the fact that the first-rank treatment strategy is still unavailable, patients often receive multimodal therapy, including palliative care, combination chemotherapy, external beam radiation, systemic therapy, and tumor debulking surgery. However, it is unfortunate that in spite of the fact that improvements are being made in each part of multimodal therapy, ATC's prognosis and recurrent disease's prevention remain unsatisfying; in the last three decades, the survival rate of ATC patients has continued to be the same. For the sake of developing effective therapeutic interventions, comprehension of the molecular mechanisms of ATC is in urgent need [28].

RETRACTED

Integrated bioinformatics analysis that places emphasis on survival analysis, network-based hub node discovery, and differentially expressed molecule screen has been put into extensive use for the purpose of identifying possible biomarkers that are linked to the prognosis, treatment, and diagnosis of ATC [29]. Thanks to the advance in gene-sequencing technology, many DEGs have been identified in some other types of tumors (such as gastric and colorectal carcinoma as well as breast carcinoma) [30]. It is possible that DEGs are functional in some aspects in diseases' occurrence and development, such as the regulation of protein expression, transcription, and posttranscriptional processing. For example, Liu et al. screened out DEGs in gastric carcinoma tissues as well as the ones that were in normality through performing multiple gene expression profile datasets' analysis by synthesis; then determination of the key genes associative with gastric cancer's prognosis and pathogenesis was obtained through conducting the analysis of the protein interaction network and Cox proportional risk model. This research is carried out with the purpose of identifying the DEGs that is pivotal in gliomas' occurrence and malignant process and the ones that are possible to be taken as ATC's molecular markers as well as therapeutic targets [31].

This research manifested that 1063 DEGs were recognized to be DEGs between ATC, and samples in normality were recognized, which were made up by 616 of downregulation as well as 447 of upregulation. Functional enrichment analysis helped to draw a conclusion that DEGs of upregulation were primarily found in organization of extracellular structure and extracellular matrix, as well as nuclear division; DEGs of downregulation significantly implicated in the thyroid hormone metabolic process and generation as well as cellular modified amino acid metabolic process. The KEGG pathway analysis displayed that there was a marked enrichment of those thyroid hormone synthesis, transcriptional misregulation in cancer, signaling pathway of p53, and PI3K-Akt. A great number of studies presented an illustration that carcinogenesis was capable of having a very strong link to thyroid hormone synthesis and transcriptional regulation. Our discoveries about functional enrichment analysis are in accordance with those of Landa et al. Landa et al demonstrated that compared to poorly differentiated thyroid cancer (PDTC), a greater mutation burden existed in ATCs, with TERT promoter's mutations' greater frequency, TP53, PI3K/AKT/mTOR pathway effectors, histone methyltransferases, and SWI/SNF subunits being included [32]. It is suggested that ATC may have a more extensive genome mutation than PDTC and cause greater virulence and higher mortality. Then we used the PPI network analysis as well as the WGCNA analysis for the purpose of determining the protein-protein interaction as well as gene coexpression modules associated with ATC's clinical characteristics. We also identified 10 hub genes (CXCL8, CDH1 AURKA, CCNA2, FN1, CDK1, ITGAM, CDC20, MMP9, and KIF11) in the PPI network. More coincidentally, except for CDH1, they are all upregulated genes in ATC. Interestingly, Hu et al. screened AURKB, CCNA2, BUB1, CDK1, CCNB1, TOP2A, AURKA, CDC20, BUB1B, and MAD2L1 as hub genes through the degree algorithm, the result of which indicated a strong correlation with other node proteins. The gene chip GSE53072, GSE65144, and GSE9115 they used contained 21 normal thyroid samples and 22 ATC samples [8]. However, a selection was completed of the top 10 DEG whose degree and betweenness algorithm are more than 4-fold of the corresponding median values as the candidate hub genes. Therefore, the hub genes screened by our algorithm are more reliable.

RETRACTED

Progress that has been made in the recent time reveals there was a pivotal part played by CXCL8 as well as their cognate receptors in inflammation that is associative with cancer and progression that is related to cancer [33, 34]. CDH1 is importantly functional in epithelial cell adhesion and participates in tumor invasion and metastasis [35]. There is an implication of AURKA and CDK1 in regulating mitosis, cell cycle progression, and a key number of oncogenic signaling pathways in a number of tumors that were in vicious condition in which neuroblastoma is included [36]. CDK1 is significant not only for cell viability but also for a great number of biological events, in which DNA damage repair, checkpoint activation, and cell cycle control can be given as examples. As a new oncogene, CCNA2 is crucial for the regulation of tumor cell growth and apoptosis [37]. There is a part played by FN1 in cell migration and adhesion, including wound healing, embryogenesis, host defense, coagulation, metastasis, and other biochemical processes [38]. It is likely that ITGAM and MMP9 participate in the process, transcriptional misregulation, and limbic system development in the cancer pathway [39]. CDC20 being aberrantly expressed is linked to diverse cancers in terms of malignant progression as well as poor prognosis [40]. KIF11 is a kind of molecular kinesin, the overexpression of which is displayed in many cancer cells, which is essential for mitosis [41].

RETRACTED

In our study, 13653 genes (the first 25% of total genes that have the greatest variance) that were taken as the input data set of WGCNA were selected for avoiding easily obtaining positive results. The WGCNA analysis showed that 4 coexpressed gene modules have expression pattern that was strongly associative, and gene ontology was used for exploring the potential biological process related to ATC. In the turquoise module, DEGs were found to be assembled in urogenital system development, ossification, and extracellular structure organization. In the grey module, DEGs were found to be gathering in the catabolic process of organic acid, small molecule, and carboxylic acid. In the blue module, an enrichment of DEGs was discovered in the organelle fission as well as in organization of extracellular structure and extracellular matrix. In the brown module, an enrichment of DEGs was found in the activation process of T cell as well as the regulation of it and lymphocyte activation. In addition, a discovery was made that these models participated in the common pathways related to ATC, including the signaling pathway of p53, PI3K/Akt, and Hippo signaling, and ECM-receptor interaction. Furthermore, we used TCGA THCA data and GSE53072 to further verify the hub gene and hub pathway. These results indicate that these hub genes and hub pathway can distinguish ATC and noncancerous samples and are likely to be candidates for early diagnostic biomarkers.

To conclude, through the performance of diverse bioinformatics analysis, nine hub genes as well as nine hub pathway genes that are possibly associative with ATC's progress were identified, and they are likely to play a role as biomarkers to assist early diagnosis and therapeutic of ATC. Nevertheless, subsequent experimental studies are in urgent demand for validation of our analysis outcome on account that our research was carried out according to analysis of data.

## Figures and Tables

**Figure 1:** Sample clustering and recognition of differentially expressed genes (DEGs) in ATC tissues. (a) Heat map's construction was completed utilizing the top 100 DEGs on the basis of fold change. (b) All DEGs' volcano plot.

**Figure 2:** DEGs' GO analysis. (a) Upregulated DEGs with fold change > 2. (b) Downregulated DEGs with fold change < −2.

**Figure 3:** KEGG enrichment analysis of all DEGs with |fold change| > 2. All DEGs were analyzed by KEGG enrichment. Fold change > 2 was taken as a cut-off value.

**Figure 4:** PPI network's module analysis. (a) Module rank 1. (b) Module rank 1's GO enrichment analysis. (c) Module rank 2. (d) Module rank 2's GO enrichment analysis. (e) Module rank 3. (f) Module rank 3's GO enrichment analysis.

RETRACTED

**Figure 5:** Determination of soft-thresholding power in the weighted gene coexpression network analysis (WGCNA). (a) Analysis of scale-free fit index for diverse soft-thresholding powers (*β*). (b) Analysis of mean connectivity for diverse soft-thresholding powers. (c) Dendrogram of all DEGs clustered on the basis of a dissimilarity measure (1-TOM).

**Figure 6:** 4 gene modules' GO enrichment analysis. (a) Turquoise module, (b) grey module, (c) blue module, and (d) brown module.

**Figure 7:** 4 gene modules' KEGG pathway enrichment analysis. (a) Turquoise module, (b) grey module, (c) blue module, and (d) brown module.

**Figure 8:** Hub genes validation using TCGA THCA (based on the GEPIA database). (a) CXCL8, (b) CDH1, (c) AURKA, (d) CCNA2, (e) FN1, (f) CDK1, (g) ITGAM, (h) CDC20, (i) MMP9, and (j) KIF11.

**Figure 9:** Hub genes validation by microarray GSE53072. (a) CXCL8, (b) CDH1, (c) AURKA, (d) CCNA2, (e) FN1, (f) CDK1, (g) ITGAM, (h) CDC20, (i) MMP9, and (j) KIF11.

## Data Availability

The data used to support the findings of this research can be obtained from the corresponding author upon request.

## Supplementary Materials

Supplementary 1 Microarray data identified 1063 genes in all as differentially expressed genes (DEG).

Supplementary 2 PPI network of overlapping DEGs constituted by 706 nodes and 6126 edges.

Supplementary 3 The cytoHubba Network Analyzer plug-in from the Cytoscape software selected top 10 DEGs whose degree and betweenness being above fourfold of the corresponding median values as the candidate hub genes.

Supplementary 4 PPI network's module analysis.

Supplementary 5 Signal paths of the KEGG pathway enrichment analysis modules 1, 2, and 3.
